RETRACTED

# *Sedum sarmentosum* Bunge extract ameliorates lipopolysaccharide- and D-galactosamine-induced acute liver injury by attenuating the hedgehog signaling pathway via regulation of miR-124 expression

**DOI:** 10.1186/s12906-020-2873-1

**Published:** 2020-03-17

**Authors:** Li Hao, Ming-wei Liu, Song-tao Gu, Xue Huang, Hong Deng, Xu Wang

**Affiliations:** 1 Department of Emergency, Yan’an Hospital of Kunming City, Panlong District, 245 Renmin East Road, Kunming, 650051 China; 2 Department of Emergency, First Affiliated Hospital of Kunming Medical University, 295 Xichang Road, Wu Hua District, Kunming, 650032 China

**Keywords:** *Sedum sarmentosum* extract, Liver injury, miR-124, Hedgehog, Inflammatory response

## Abstract

**Background:**

*Sedum sarmentosum* is traditionally used to treat various inflammatory diseases in China. It has protective effects against acute liver injury, but the exact mechanism of such effects remains unclear. This study investigated the protective effects of *S. sarmentosum* extract on lipopolysaccharide (LPS)/D-galactosamine (D-GalN)-induced acute liver injury in mice and the mechanism of such effects.

**Methods:**

Mice were randomly divided into control, treatment, model, and model treatment groups. Acute liver injury was induced in model mice via intraperitoneal injection of LPS and D-GalN with doses of 10 μg/kg of LPS and 500 mg/kg, respectively. The mRNA expression levels of miR-124, Hedgehog, Patched (Ptch), Smoothened (Smo), and glioma-associated oncogene homolog (Gli) in liver tissues were determined through RT-PCR, and the protein levels of Hedgehog, Ptch, Smo, Gli, P13k, Akt, HMGB1, TLR4, IkB-α, p-IkB-α, and NF-kB65 were evaluated via Western blot analysis. The serum levels of IL-6, TNF-α, CRP, IL-12, and ICAM-1 were determined via ELISA. TLR4 and NF-κBp65 activity and the levels of DNA-bound NF-KB65 and TLR4 in LPS/D-GalN-induced liver tissues were also determined. We recorded the time of death, plotted the survival curve, and calculated the liver index. We then observed the pathological changes in liver tissue and detected the levels of liver enzymes (alanine aminotransferase [ALT] and aspartate transaminase [AST]) in the serum and myeloperoxidase (MPO) and plasma inflammatory factors in the liver homogenate. Afterward, we evaluated the protective effects of *S. sarmentosum* extracts on acute liver injury in mice.

**Results:**

Results showed that after *S. sarmentosum* extract was administered, the expression level of miR-124 increased in liver tissues. However, the protein expression levels of Hedgehog, Ptch, Smo, Gli, P13k, p-Akt, HMGB1, TLR4, p-IκB-α, and NF-κB65 and the mRNA expression levels of Hedgehog, Ptch, Smo, and Gli decreased. The MPO level in the liver, the IL-6, TNF-α, CRP, IL-12, and MMP-9 levels in the plasma, and the serum ALT and AST levels also decreased, thereby reducing LPS/D-GalN-induced liver injury and improving the survival rate of liver-damaged animals within 24 h.

RETRACTED

**Conclusions:**

*S. sarmentosum* extract can alleviate LPS/D-GalN-induced acute liver injury in mice and improve the survival rate of mice. The mechanism may be related to the increase in miR-124 expression, decrease in Hedgehog and HMGB1 signaling pathway activities, and reduction in inflammatory responses in the liver. Hedgehog is a regulatory target for miR-124.

## Background

Liver injury has become an increasingly serious problem worldwide. In Western countries, the incidence of acute liver injury caused by alcohol, drugs, and other factors increases annually [1]. A recent study revealed that in China, most cases of drug-induced liver injury (DILI) present hepatocellular injury (51.39%), followed by mixed injury (28.30%) and cholestatic injury (20.31%) [2]. The leading single classes of implicated drugs were determined to be traditional Chinese medicines or herbal and dietary supplements (26.81%) and antituberculosis medication (21.99%) [2]. Chronic DILI occurred in 13.00% of the cases. Out of the 44.40% of hepatocellular DILI cases that matched Hy’s law criteria, only 1.08% or 280 cases progressed to hepatic failure, 0.01% or two cases underwent liver transplantation, and 0.39% or 102 patients died. A total of 23.38% of the patients with DILI had combinations of viral hepatitis, fatty liver, and other basic liver diseases, and these patients had more severe liver damage and higher risk of liver failure and death than the other patients [2]. The same study also showed that the annual incidence of DILI in the general population of China is at least 23.80/100,000, which is higher than the value reported in Western countries [2]. Traditional Chinese medicines, herbal and dietary supplements, and antituberculosis drugs are the leading causes of DILI in mainland China [2].

People generally avoid using drugs that can cause liver damage because no specific treatment is available for drug-induced liver damage. Many active ingredients in traditional Chinese medicine protect the liver from toxic injury and reduce liver tissue damage and the degree of such damage. These active ingredients include polyphenolic compounds, flavonoids, saponin compounds, organic acid compounds, terpenoids, phenylpropanoids, sugars, and alkaloids [3]. *Sedum sarmentosum* Bunge (SSB), also known as *Sedum sarmentosum* (SS), has extracts that exert preventive and protective effects on alcohol-induced liver injury [3], but the mechanism remains unclear, and further research is required. SSB is a fresh or dry whole grass that is used to relieve jaundice symptoms, clear heat, and remove toxicity. As a commonly used Chinese medicinal plant, *SS* is primarily utilized to treat jaundice with damp-heat pathogen and difficulty in urination [4]. The main components of *SS* are flavonoids, amino acids, sugars, proteins, and triterpenoids, which have good biological activity. For example, the water-soluble total glycosides of *Trifolium* and *Pennisetum* have good immunomodulatory effects and can enhance muscle strength, decrease enzyme activities, and protect liver functions [4]. The total flavonoids of *SS* exert antitumor effects [5], and alkaloids have liver-protecting effects. The main active components in the decoction of SS are water-soluble total glycosides and total flavonoids; among these components, wheat flavin-7-0-β-D-glucoside has liver protection effects as verified by pharmacological studies, and the less stable total flavonoids, such as aglycone, can inhibit the release of inflammatory mediators, repair damaged liver cells, and significantly improve liver functions (i.e., significant effects on alanine aminotransferase [ALT]) [6]. However, the mechanism of such effects remains unclear and requires further study.

RETRACTED

Intraperitoneal injection of D-galactosamine (D-GalN) and lipopolysaccharide (LPS) is a convenient method of constructing model mice with acute liver injury [7]. LPS, a major component of endotoxins secreted by Gram-negative bacteria, causes apoptosis and necrosis of hepatocytes by stimulating the release of inflammatory factors from immune cells, including macrophages [7]. D-GalN inhibits the synthesis of biomacromolecules, such as RNA and protein, by consuming uridine triphosphate in the liver, thereby causing liver inflammation and diffused necrosis of hepatocytes [7, 8]. The synergistic effect of LPS and D-GalN causes the liver cells of experimental animals to die within a short time, and the liver physiological function becomes seriously impaired. The mechanism of liver injury caused by endotoxins is closely associated with oxidative and endotoxin-mediated inflammatory responses, but effective treatment remains lacking [9].

The Hedgehog signaling pathway is primarily composed of extracellular Hedgehog signaling protein, specific receptor Patched (Ptch) on the surface of cell membranes, Smoothened (Smo) transmembrane proteasome, and nuclear transcription factor Gli (glioma-associated oncogene homolog) [10]. The increased expression of Ptch, which is the main target gene and an important component of the Hedgehog signaling pathway, is often considered a marker of Hedgehog signaling pathway activation [10]. The Hedgehog ligand can be identified using Smo after binding to the Ptch receptor present on the cell membrane. Smo is a transmembrane protein that can activate the intracellular signaling pathway. After the transcription factor (Gli) in the cytoplasm is activated, it enters the nucleus and regulates the transcription of target genes [11]. Many studies have reported that the Hedgehog signaling pathway may be involved in acute inflammatory responses in tissues through the regulation of inflammatory factors [12, 13]. Dunaeva et al. found that the Shh protein is a potent monocyte chemotactic factor and can activate other classical signaling pathways [14], such as PI3K and HMGB1, thereby allowing inflammatory cells to migrate.

RETRACTED

MicroRNAs (miRNAs) are a class of small non-coding RNAs in eukaryotes with approximately 18–21 nucleotides. Most miRNAs identify the 3′-untranslated regions (3′-UTRs) of the mRNA molecules of corresponding target genes through complete or partial base complementarity, inhibit the expression of the target genes at the post-transcriptional level, or cause mRNA degradation. miRNAs are often highly conserved and tissue-specific, and their normal physiological functions are affected when they are mutated or abnormally expressed. miRNAs are involved in various biological processes, including cell proliferation, differentiation, inflammatory immune regulation, tissue and organ development, apoptosis, hormone secretion, fat metabolism, and various liver disease-related pathophysiological processes [15–17]. Certain miRNAs, including miR-146, miR-155, miR-200, miR-21, miR-16, miR-130, and miR-124, are associated with acute inflammatory diseases [16]. These miRNAs are closely involved in various inflammation-related diseases by regulating the expression of target genes, which play important roles in inflammation-related pathways. Thus, miRNAs have become new targets for the treatment of inflammation-related diseases. However, the regulatory mechanism of miRNAs in inflammation is still unclear and must be further studied.

Increasing the miR-124 expression in human aortic valve cells can inhibit the activities of IκBκB and NF-κB signaling pathways [18]. miR-124 can regulate the occurrence and development of pancreatic cancer by regulating Hedgehog target signaling [19]. Previous studies have found that SS prevents D-GalN/LPS-induced fulminant hepatic failure, and this protection is likely associated with SS’ anti-apoptotic activity and the down-regulation of mitogen-activated protein kinase activity associated at least in part with the suppressed transcription of LPS receptors [6]. SSB extract ameliorates tilapia fatty liver via PPAR and P53 signaling pathways [3]. In the current study, we hypothesized that miR-124 regulates the occurrence and development of D-GalN/LPS-induced acute liver injury by regulating the Hedgehog signaling pathway. We determined if SS extract can regulate the effects of miR-124 on D-GalN/LPS-induced acute liver injury to reveal the protective mechanism of SS in the treatment of acute liver injury.

RETRACTED

## Methods

### SSB extract preparation

SSB (cat. no. YYR336; Shaanxi Yongyuan Biotechnology Co., Ltd., Shaanxi, China) was extracted in accordance with a previously described method [20]. SSB (82.50% purity) was purchased from Xi’an Yuze Biological Technology Co., Ltd. (Xi’an, China) and identified by Professor Yi Fu at the Department of Pharmacognosy, Yunnan Chinese Medical University. Approximately 500 g of SSB crude material was subjected to extraction and purification procedures. Crushed powder was added to 4 L of 70% (v/v) ethanol and extracted twice for 2 h with refluxing. The extracts were evaporated using a rotary evaporator then filtrated and concentrated. The drugs of the refluxing extract needed further refluxing, filtration, and concentration. For animal experiments, 1 g of SSBE was dissolved in 10 ml of normal saline, resulting in a final concentration of 100 mg/ml.

### High-performance liquid chromatography (HPLC) analysis of SSB extract

Quercetin, kaempferide, and isorhamnetin, which have been reported as components of SSB that inhibit acute liver injury [4], were used as standard substances to detect the effects of different solution fractions of ethanol extract from SSB. The main active ingredients of the SSB extract were determined through HPLC. An e2695 high-performance liquid chromatograph with a 2998 diode array detector and an Empower chromatography workstation (Waters, USA) was used to determine the contents of quercetin, kaempferide, and isorhamnetin. The chromatographic conditions were chromatographic column, Hedera ODS-2 (4.6 mm × 200 mm, 5 m); mobile phase, acetonitrile (A): 0.1% phosphoric acid solution and (B) gradient elution (Table 1); detection wavelength of 310 nm; flow rate of 0.8 ml/min; column temperature of 35 °C; and injection volume of 10 μl. Three compounds were identified through a comparison of the peak value of sample retention time. The content of each compound in the SSB extract was determined with an external standard method. Each HPLC run was repeated three times.

**Table 1:** Gradient Elution Procedure

t/min	A∶B
0 → 10	10∶90
10 → 30	10∶90 → 15∶85
30 → 50	15∶85 → 25∶75
50 → 60	25∶75 → 40∶60
60 → 75	40∶60 → 70∶30
75 → 80	70∶30 → 10∶90

RETRACTED

### Cell culture, transfection, and grouping

Rat hepatocyte–Kupffer cells (KCs) were purchased from Bioleaf Biotech Inc. (Shanghai, China) and cultured in an L-15 medium mixture containing 2% penicillin/streptomycin, 10% fetal bovine serum, and DMEM medium at 37 °C and 5% CO_2_. The experiment was conducted when the cells reached the logarithmic growth phase. The rat hepatocyte–KCs were transfected with miRNA mimics, an inhibitor of miR-124, and NC by using Lipofectamine 2000 as a transfection reagent then labeled as the miR-124 experimental group (mimitics), inhibitory group (inhibitor), and control group (NC), respectively. After 24 h of transfection, the cell growth inhibition rate was detected using an MTT kit. Total RNA and protein were determined for quantitative real-time polymerase chain reaction (qRT-PCR) and Western blot analysis.

The cells were synchronized for 24 h and grouped after reaching 60% confluency. To observe the effects of baicalin on the inflammation and proliferation of LPS-induced rat hepatocyte–KCs, the cells were divided into the following groups: normal control, LPS induced, LPS plus low-dose (1 g/l) SSB extract, LPS plus medial-dose (2 g/l) SSB extract, and LPS plus high-dose (2.5 μmol/l) SSB extract. Different concentrations of SSB extract in the range of 25–75 μM were added to the 2 h cell culture, and 1.0 mg/L of LPS solution was added after 2 h. The cultures with SSB extract were incubated for another 24 h. Subsequently, various related indicators were measured.

### MTT cell proliferation assay

Cell proliferation in all groups was analyzed using an MTT assay kit (KeyGen Biotech Inc., Nanjing, China). Briefly, the cell medium was discarded, and the cells were incubated with 90 μL of FBS-free medium and 20 μL of MTT at 37 °C for 4 h. Then, the cells were treated with 150 μL of DMSO for 10 min. The optical density (OD) was determined with a microplate reader at 490 nm wavelength. Three wells were prepared for each group. Cell proliferation inhibition rate was calculated using the following formula: cell proliferation inhibition rate (%) = (OD value in control group−OD value in experimental group)/OD value in control group× 100%. IC50 was calculated with the Bliss method as previously described [21].

### Dual-luciferase activity assay

Target Scan (http://www.targetscan.org) was used to determine possible miR-124 targets. Rat hepatocyte–KCs (1 × 10^5^) were cultured on 24-well plates and transfected using Lipofectamine 2000 (Invitrogen, Carlsbad, CA, USA) with one of the following: SHH-3′UTR-wt, SHH-3′UTR-mt, miR-124, or mi-NC. The rat hepatocyte–KCs were lysed after transfection for 24 h, and the gene expression of the luciferase reporter was detected with the Dual-Luciferase Reporter Assay System Kit in accordance with the manufacturer’s instructions. Approximately 100 μL of 1× cell lysate was added to each well, and the plate was shaken slowly for 15 min at room temperature. Then, 10 μL of cell lysate was added to 50 μL of luciferase assay reagent II, and the solution was mixed and firefly luciferase activity was measured with a fluorescence luminometer. Approximately 50 μL of Renilla fluorescein reagent was added to detect Renilla luciferase activity. The relative activity ratio of firefly and Renilla luciferase fluorescence activity was used as the reporter gene activity (the Renilla luciferase fluorescence value was utilized as the internal reference).

RETRACTED

### Animals

After obtaining animal care approval from the Laboratory Animal Care and Use Committee of Kunming Medical University (Kunming, China), experiments were performed on six-week-old male C57BL/6 mice (12 ± 3.4 g body weight, Kunming Medical University Laboratory Animal Center, Kunming, China). The mice were kept under conditions that conformed to the National Institutes of Health’s Guide for the Care and Use of Laboratory Animals and Animal Care Committee of Kunming Medical University. All mice were maintained on a standard diet and given water ad libitum at 12 h day and night cycles. The animals did not undergo fasting prior to the procedure. Anesthesia was administered by a consultant anesthesiologist who had been specially trained in providing rodent anesthesia.

### Preparing the inducer of acute liver injury

Acute liver injury in mice was induced using LPS/D-Gal as previously reported [22]. Briefly, mice were intraperitoneally injected with 10 μg/kg of LPS and 500 mg/kg of D-Gal to induce acute liver injury for 6 h. Successful modeling was confirmed via a pathological examination.

### Animal therapies

Forty mice were randomly divided into five groups, namely, normal, normal treatment, model normal, model treatment, and silymarin, with eight mice per group. In Group 1 (normal group), the mice were treated with the same amount of normal saline (5 ml/kg) via the tail vein. In Group 2 (normal treatment group), the mice were injected once a day with SSB extract (100 mg/kg) via the tail vein. In Group 3 (model normal group), acute liver injury was induced in mice by intraperitoneal injection of LPS (10 μg/kg) and D-Gal (500 mg/kg). In Group 4 (model treatment group), after acute liver injury was induced, SSB extract (100 mg/kg) was injected into the mice once a day via the tail vein. In Group 5 (silymarin group), the acute liver injury-induced mice were injected with silymarin (200 mg/kg) once a day via the tail vein as described previously [23]. The mice were made to undergo fasting but were given a normal dose of water. After intraperitoneal injection of LPS (10 μg/kg) plus D-Gal (500 mg/kg) for 24 h, the mice were narcotized with 0.2% sodium pentobarbital (60 mg/kg, Sigma-Aldrich; Merck Millipore, Darmstadt, Germany) and sacrificed via cervical dislocation. Blood was obtained from the eyelids, stored at room temperature for 2 h, and centrifuged at 4 °C and 4000 r/min for 10 min to collect the serum. The collected serum was stored in a refrigerator at − 20 °C for examination. The abdominal cavity of a mouse was immediately cut, and the same part of the liver tissue was collected, fixed with 10% formaldehyde solution, and dehydrated with gradient ethanol. The liver tissue samples were embedded with paraffin, routinely sliced, and stained with hematoxylin–eosin (HE). Changes in the liver pathological morphology of the mice in each group were observed using a light microscope.

RETRACTED

### Intravenous tail administration of AdCMV-miR-124

A constitutively active miR-124 expression construct was delivered to the mice through intravenous tail administration of 1 × 10^9^ pfu AdCMV-miR-124 for 14 d in accordance with a previously described method [24]. The expression of miR-124 in liver tissue was amplified by RT-PCR, which confirmed that liver miR-124 overexpression was successful. We then induced acute liver injury in the mice by intraperitoneal administration of LPS and D-GalN for 24 h. The control mice received an empty adenoviral vector on the same schedule. The mice were then narcotized with 0.2% sodium pentobarbital (Sigma-Aldrich; Merck Millipore, Darmstadt, Germany) and sacrificed via cervical dislocation. Blood was obtained from the eyelids, stored at room temperature for 2 h, and centrifuged at 4 °C and 4000 r/min for 10 min to collect the serum. The collected serum was then stored in a refrigerator at − 20 °C for examination. The abdominal cavity of a mouse were cut immediately, and the same part of the liver tissue was collected, fixed with 10% formaldehyde solution, and dehydrated with gradient ethanol. The samples were embedded with paraffin, routinely sliced, and stained with HE. Changes in the liver pathological morphology of the mice in each group were observed with a light microscope.

### Real-time PCR

Total RNA was extracted from liver tissue with the TRIzol method. A reverse transcription kit (TaKaRa, Japan) was used for the reverse transcription of RNA samples to synthesize cDNA. Reverse transcription was carried out at 37 °C for 15 min, and the inactivation of reverse transcriptase was performed at 85 °C for 15 s. RT-qPCR was performed with SYBR Premix Ex Taq™ Real-Time PCR Kit (TaKaRa, Japan). PCR was conducted by activating DNA polymerase at 95 °C for 5 min. The reaction system comprised 5.0 μL of 5× SYBR green fluorescent dye, 3.4 μL of DEPC water, 0.2 μL of upstream and downstream primers, 1.0 μL of the DNA sample, and 0.2 μL of ROX. Then, 40 cycles of two-step PCR (95 °C for 10 s and 60 °C for 30 s) were performed, and the final extension time was at 75 °C for 10 min, which was maintained at 4 °C. The primer concentration is 10 μM. All primers were obtained from Genewiz (Jiangsu, China). RNA expression was analyzed using the 2^−∆∆Ct^ method [25]. β-actin and U6 were used as the internal references for mRNA and miRNA, respectively. The primer sequence and product size of the gene are shown in Table 2.

RETRACTED

**Table 2:** Gene primer sequences for RT-PCR analysis

miR-124	F-5′-GAATCCCATCGCGTTCCCCAAACCCC-3′	77 bP
	R-5′-GGATTCAGGGATGAAGGTGCTGGCCT-3′	
U6	**F-5′-CTCGGCTCGGCAGCACA-3′**	**93 bP**
	**R-5′-ACGCTTCACGAATTTGCGT-3′**	
SHH mRNA	**F-5′-CTCGTGCTACGGAGTCATCG-3′**	**158 bP**
	**R-5′-CCTCGCTTCCGCTACAGATT-3′**	
Ptch mRNA	**F-5′-AAAGAACTGCGGCAAGTTTTTG-3′**	**254 bP**
	**R-5′-CTTCTCCTATCTGACGGGT-3′**	
Smo mRNA	**R-5′-ATGATGGACCTGTTGCG-3′**	**142 bP**
	**R-5′-GTTGGCTTGTTCTTCTGG-3′**	
Gli mRNA	**R-5′-TTCTTCTGCTGACACTCTGGGATA-3′**	**251 bP**
	**R-5′-CCTCAAGTCGAGGACACTGGTTA-3′**	
Akt mRNA	**F-5′-TCACCTCTGAGACCGACACC-3′**	**236 bP**
	**R-5′-ACTGGCTGAGTAGGAGAACTGG-3′**	
P13K mRNA	**F-5′-TGGTACATATCGGGCTAGAAG-3′**	**185 bP**
	**R-5′-CCATACTGTACCAGGCAAGGT-3′**	
β-actin	**5′-GTTGGCTT-GTTCTTCTGG-3′**	**298 bP**
	**5′-GCTGCCTCAACACCTCAACCC-3′**	

### Western blot assays

Total protein was extracted from rat liver by using the strong RIPA protein lysis method and lysed on ice for 45 min. The lysis fluid was mixed at intervals during lysis and centrifuged at 4 °C and 14,000 g for 15 min. The supernatant was collected after lysis. Protein concentration was determined using the bicinchoninic acid disodium method, and the concentration in each group was adjusted for consistency. Sodium dodecyl sulfate–polyacrylamide gel electrophoresis (10% separating gel and 5% stacking gel) was carried out. Protein was transferred to the cellulose nitrate membrane via electrorotation, which was sealed with 5% skim milk powder for 1 h. Afterward, it was added with diluted primary antibodies overnight at 4 °C (SHH [1:1000], Ptch [1:1000], Smo [1:1000], p-IkB-α [1:1000], TLR4 [1:1000], Akt [1:1000], p-Akt [1:1000], IkB [1:1000], NF-kB65 [1:1000], p-NF-kB65 [1:1000], B-actin [1:1000] and HMGB1 [1:1000]) (Abcam, Cambridge, UK) in accordance with the manufacturer’s instructions. Thereafter, rabbit anti-rat IgM antibody (Abcam, Cambridge, UK) was added after washing with TBST, and the samples were incubated at room temperature for 2 h. The film was washed, and the color was developed using enhanced chemiluminescence. Furthermore, images were collected by an automatic gel imager, and Image J software was used for strip analysis. The relative expression of the target protein was expressed as the ratio of the target protein to the gray value of the internal reference β-actin band.

RETRACTED

### Detection of NF-kB65 and TLR4 protein expression by immunohistochemistry

The liver tissue sections were dewaxed, hydrated, given antigenic hyper repair, blocked with 5% BSA at 37 °C for 30 min, added with primary antibody (NF-kB65 78:1:250; TLR4: 1:50), and incubated at 4 °C overnight. After incubation, the liver tissue sections were washed three times (5 min each time) with PBS buffer. Then, secondary antibody was added, and further incubation at 37 °C for 30 min was performed. The tissue sections were stained with DAB after PBS washing, counterstained with hematoxylin for 45 s, dehydrated, made transparent, sealed, and photographed. The absorbance ratio was analyzed using Image Pro Plus 6.0 software.

### Myeloperoxidase (MPO) enzyme activity assay

The presence of MPO was used as an index of neutrophil accumulation in the liver [26] and determined using an MPO colorimetric assay kit (BioVision, Milpitas, CA, United States) according to the manufacturer’s instructions.

### Enzyme-linked immunosorbent assay (ELISA)

The concentrations of cytokines in the serum, cell, and liver tissue supernatant were determined by ELISA for mouse IL-6, TNF-а, CRP, IL-12,MMP-9, DNA-bound NF-KB65, and TLR4 (eBioscience, San Diego, CA) according to the manufacturer’s instructions.

### Measurement of alanine aminotransferase (ALT) and aspartate aminotransferase (AST)

After intraperitoneal injection of LPS (10 μg/kg) and D-Gal (500 mg/kg) for 24 h, blood was obtained from the venous plexus and centrifuged (603×g) for 10 min. ALT and AST levels in the serum were measured with an automated biochemical clinical analyzer (Hitachi, Tokyo, Japan) according to the manufacturer’s instructions.

### Histological analysis

The mice were euthanized after orbital blood was obtained. The liver tissue was fixed in 4% neutral formalin solution, embedded in paraffin, and cut into 4 mm thick sections. The tissue was dewaxed and stained with HE. A light microscope (× 200) was used to observe histopathological changes in the liver. The damage scores were estimated by counting the morphological alterations in 10 randomly selected microscopic fields from six samples of each group and from at least three independent experiments. The morphological liver integrity was graded on a scale of 1 (excellent) to 5 (poor). Liver damage scores was adopted from the study of t’Hart et al. [27] and described in Table 3.

RETRACTED

**Table 3:** Liver damage pathological score and scoring criteria

Liver damage scores	Histological changes
1	normal rectangular structure
2	rounded hepatocytes with an increase in sinusoidal spaces
3	vacuolization
4	nuclear pyknosis
5	necrosis

### Survival rate analysis

The methods used for the analysis of survival rate was based on a previous study [28]. A total of 75 mice were divided into five groups (15 mice/group): control, control SSB, model, model SSB, and model silymarin. The aim was to observe the survival rate. The treatment method was similar to that mentioned above. Observations began upon treatment with SSB extract, and endpoints were set at 120 h after treatment.

### Statistical analysis

SPSS 19.0 was used to analyze the data. Data were expressed as mean ± standard deviation. The significance was determined using two-tailed Student’s t-test or one-way analysis of variance with Bonferroni post-tests when applicable. *P* < 0.05 indicates a significant difference between two groups.

## Results

### Main active chemical components of SSB by HPLC analysis

HPLC analysis indicated that 1 g of SSB contained 0.93 mg of quercetin, 0.34 mg of kaempferide, and 0.27 mg of isorhamnetin. Quercetin was the major component (Fig. 1).

**Fig. 1:** Chromatogram of the chemical reference substances and sample. **a**. Chromatogram of the chemical reference substances. **b**. Chromatogram of various samples: 1, Quercetin; 2, Kaempferide; 3, Isorhamnetin

### Effect of miR-124 on hedgehog, Ptch, Smo, Gli, Akt, p-IkB-а, NF-kB65, and inflammatory medium in rat hepatocyte–KCs

The expression levels of Hedgehog, Ptch, Smo, Gli, Akt, p-IkB-а, and NF-kB65 in miR-124 mimic, control miR-124 mimic, miR-124 inhibitor, and control miR-124 inhibitor were measured using Western blot analysis 24 h after transfection with Lipofectamine 2000. As shown in Fig. 2, increased miR-124 levels significantly decreased Hedgehog, Ptch, Smo, Gli, Akt, p-IkB-а, and NF-kB65 expression, suggesting that miR-124 may regulate the Hedgehog inflammatory signaling pathway (Figs. 2 a–e). To further analyze the effect of miR-124 on the inflammatory medium in rat hepatocyte–KCs, the levels of IL-6 and TNF-а in these cells were measured by ELISA. As shown in Fig. 2, increased miR-124 levels significantly decreased IL-6 and TNF-а production (Fig. 2 f and g).

**Fig. 2:** Effect of miR-124 on the Hedgehog signaling pathway, inflammatory response, and cell proliferation inhibition rate in rat hepatocyte–KCs. (**a** and **b**) qRT-PCR analysis of miR-124 levels in rat hepatocyte–KCs transfected with control mimic, miR-124 mimic, control inhibitor, or miR-124 inhibitor for 24 h. (**c** and **d**) Quantitative Western blot analysis of Hedgehog, Ptch, Smo, Gli, Akt, p-IkB-а, and NF-kB65 protein levels in rat hepatocyte–KCs transfected with control mimic, miR-124 mimic, control inhibitor, or miR-124 inhibitor for 24 h. (**e** and **f**) Levels of IL-6 and TNF-а in rat hepatocyte–KCs with control mimic, miR-124 mimic, control inhibitor, or miR-124 inhibitor for 24 h. Data are expressed as mean ± SD of three independent experiments. *P < 0.05: versus control mimic; #*P* < 0.05: versus control inhibitor

RETRACTED

### Effect of miR-124 on cell proliferation inhibition rate in rat hepatocyte–KCs

The inhibition rate of cell proliferation in rat hepatocyte–KCs by miR-124 was detected using MTT assay. As shown in Fig. 3, increased miR-124 levels significantly decreased the inhibition rate of cell proliferation in rat hepatocyte–KCs. Meanwhile, the influence of different concentrations of miR-124 inhibitor in the range of 25–100 nM on the hepatocyte–KCs’ proliferation inhibition rate and IC50 was investigated. Twenty-four hours after the transfection of miR-124 inhibitors, the proliferation inhibition rate of hepatocyte–KCs was detected by MTT assay, and IC50 was calculated with the Bliss method. Different concentrations (25–100 nM) of the miR-124 inhibitor increased the proliferation inhibition rate of hepatocyte–KCs in a concentration-dependent manner. The concentration of the miR-124 inhibitor was 64.8 nM for IC50.

**Fig. 3:** Effect of miR-124 on hepatocyte–KC proliferation inhibition rate and IC50. Control mimic, miR-124 mimic, control inhibitor, or miR-124 inhibitor was transfected for 24 h. Cell proliferation inhibition rate and IC50 were measured. Data are expressed as mean ± SD of three independent experiments. *P < 0.05: versus control mimic; #*P* < 0.05: versus control inhibitor

### Hedgehog was a direct target of miR-124

We used a well-known database to predict miR-124 targets and found that SHH, an important pro-inflammatory regulator of inflammation-related liver injury, was a candidate miR-124 target. Overexpressing miR-124 considerably reduced SHH mRNA and protein levels (Fig. 4 a and b). To further confirm the interaction between SHH and miR-124, we built SHH-3′UTR-wt and SHH-3′UTR-mt constructs for dual-luciferase reporter assay (Fig. 4 c and d). As expected, miR-124 bound with SHH-3′UTR-wt but not the mutant version (Fig. 4 d).

**Fig. 4:** SHH is a miR-124 target. **a** SHH mRNA levels decreased in miR-124-overexpressing rat hepatocyte–KCs (*P* < 0.05). **b** Overexpressing miR-124 in rat hepatocyte–KCs decreased SHH protein levels compared with that of vector controls (*P* < 0.05). **c** MiR-124 bound to SHH-3′UTR-wt, but the binding was blocked by SHH-3′UTR-mt. **d** Dual-luciferase reporter assays confirmed that miR-124 mimic bound to SHH-3′UTR-wt but not the mutated form (*P* < 0.05)

RETRACTED

### Overexpressing miR-124 decreased LPS/D-GalN-induced acute liver injury and liver damage scores in mice

The Hedgehog signaling pathway is involved in LPS/D-GalN-induced acute liver injury and liver damage scores in mice [12, 29]. Liver tissues from the four groups were stained with HE for histopathological analysis to further evaluate if overexpressing miR-124 decreased LPS/D-GalN-induced acute liver injury in mice. Following LPS/D-GalN exposure (Fig. 5), normal histological structures of hepatic lobules were observed in the livers of the mice in the control group (Fig. 5 a). The model group treated with LPS/D-GalN exhibited complete hepatocyte damage with hepatocellular vacuolization and focal hepatic necrosis (Fig. 5 a). Cells pretreated with 1 × 10^9^ pfu AdCMV-miR-124 showed an increased miR-124 expression (Fig. 5 b and c) and exhibited normal liver cell structures with a well-defined cytoplasm and nucleus and ribbon-like hepatocyte arrangements (Fig. 5 a).

**Fig. 5:** Overexpressing miR-124 attenuated LPS/D-GalN-induced acute liver injury and the activity of the Hedgehog signaling pathway. **a** Representative images of HE-stained liver sections from four experimental groups (magnification, × 400) after the administration of 1 × 10^9^ pfu AdCMV-miR-124 for 14 d and intraperitoneal administration of LPS and D-GalN to induce acute liver injury. **b** and **c** Representative RT-PCR showing the miR-124 expression levels in LPS and D-GalN to induce liver injury 14 d after the administration of 1 × 10^9^ pfu AdCMV-miR-124 and intraperitoneal administration of LPS and D-GalN to induce acute liver injury. **d** and **e** Representative Western blot analysis and statistical summary of densitometric analysis showing Hedgehog, Ptch, Smo, Gli, p-IkB-α, and NF-kB65 protein expression levels in liver tissue 24 h after the administration of 1 × 10^9^ pfu AdCMV-miR-124 for 14 d and intraperitoneal administration of LPS and D-GalN to induce acute liver injury. **f** Liver injury score from four experimental groups (magnification, × 400) after the administration of 1 × 10^9^ pfu AdCMV-miR-124 for 14 d and intraperitoneal administration of LPS and D-GalN to induce acute liver injury. Data are expressed as mean ± SD. *P < 0.05: compared with the control group; #*P* < 0.05 and ##*P* < 0.01 compared with the model group

We also analyzed the effect of overexpressing miR-124 on LPS/D-GalN-induced liver damage scores in mice. We measured liver damage scores as previously described [28]. The liver damage score significantly increased in the model group compared with that in the control group (*P* < 0.01) (Fig. 5 f). Cells pretreated with 1 × 109 pfu AdCMV-miR-124 showed increased miR-124 expression (Fig. 5 b and c). The liver damage score significantly decreased compared with that in the model group (*P* < 0.05) (Fig. 5 f).

RETRACTED

### Overexpressing miR-124 decreased hedgehog, Ptch, Smo, Gli, p-IkB-α, and NF-kB65 protein expression levels in LPS/D-GalN-induced acute liver injury mouse liver

To clarify the effect of overexpressing miR-124 on Hedgehog, Ptch, Smo, Gli, IkB, and NF-kB65 protein expression levels in mice with LPS/D-GalN-induced acute liver injury, Hedgehog, Ptch, Smo, Gli, p-IkB-α, and NF-kB65 protein expression levels were analyzed via Western blot analysis. As shown in Fig. 5, overexpressing miR-124 decreased Hedgehog, Ptch, Smo, Gli, p-IkB-α, and NF-kB65 protein expression levels in mice with LPS/D-GalN-induced acute liver injury (Fig. 5 d and e). Overexpressing miR-124 attenuated LPS/D-GalN-induced inflammation by regulating the Hedgehog signaling pathway.

### Effects of SSB extract on miR-124/hedgehog and NF-κB65 signaling pathways in LPS-induced rat hepatocyte–KCs

We further observed the effect of SSB extract on miR-124/Hedgehog and NF-κB65 signaling pathways in LPS-induced rat hepatocyte–KCs. Hepatocyte–KCs were incubated at various concentrations of SSB extract (1.0, 2, and 2.5 g/l) and LPS (1 mg/l) for 24 h. The miR-124 expression was measured by RT-PCR. Hedgehog, Smo, Gli, p-Akt, and NF-κB65 protein levels were measured by Western blot. As shown in Fig. 6, the SSB extract decreased the Hedgehog, Smo, Gli, p-Akt, and NF-κB65 protein levels (Figs. 6 a–c) and increased the levels of miR-124 in LPS-induced hepatocyte–KCs in a concentration-dependent manner (Figs. 6 d–e). SSB extract concentrations as low as 2.0 g/l effectively increased the miR-124 expression and blocked the activity of miR-124/Hedgehog and NF-κB65 signaling pathways in LPS-induced hepatocyte–KCs (Figs. 6 a–e).

**Fig. 6:** Effect of SSB extract on miR-124/Hedgehog and NF-κB65 signaling pathways in LPS-induced rat hepatocyte–KCs. Hepatocyte–KCs were incubated at various concentrations of SSB extract (1.0, 2, and 2.5 g/l) and LPS (1 mg/l) for 24 h. miR-124 expression was measured by RT-PCR. Hedgehog, Smo, Gli, p-Akt, and NF-κB65 protein levels were measured by Western blot. *P < 0.05 and **P < 0.01: compared with the control group; #*P* < 0.05 and ##*P* < 0.01 compared with the LPS group

### Effects of SSB extract on LPS-induced rat hepatocyte–KC inflammation

To investigate the effect of SSB extract on LPS-induced rat hepatocyte–KC inflammation, hepatocyte–KCs were incubated at various concentrations of SSB extract (1.0, 2, and 2.5 g/l) and LPS (1 mg/l) for 24 H*. IL*-6 and TNF-α in the hepatocyte–KCs were measured using ELISA. As shown in Fig. 7, the SSB extract decreased the levels of IL-6 and TNF-α in the LPS-induced hepatocyte–KCs in a concentration-dependent manner (Figs. 7 a–b). SSB extract concentrations as low as 2.0 g/l effectively decreased the IL-6 and TNF-α levels in the LPS-induced hepatocyte–KCs.

RETRACTED

**Fig. 7:** SSB extract inhibited LPS-induced rat hepatocyte–KC inflammation. Hepatocyte–KCs were incubated at various concentrations of SSB extract (1.0, 2, and 2.5 g/l) and LPS (1 mg/l) for 24 H*. IL*-6 and TNF-α in hepatocyte–KCs were measured using ELISA. Data are expressed as mean ± SD. * *P* < 0.05 and **P < 0.01: compared with the control group; #*P* < 0.05 and ##*P* < 0.01: compared with the LPS group

### Effects of SSB extract on miR-124 expression level in LPS/D-GalN-induced acute liver injury in mice

The miR-124 signaling pathway is involved in the LPS-mediated inflammatory response [30]. We observed the effects of SSB extract on the expression levels of miR-124 in LPS/D-GalN-induced mouse liver tissue. The miR-124 expression was determined via RT-PCR and in situ hybridization. As shown in Fig. 8, the expression levels of miR-124 were significantly reduced compared with those of the control group after LPS/D-GalN-induced acute liver injury in mice (Figs. 8 a–c). However, treatment with SSB extract significantly increased the miR-124 expression compared with that of the model group (Figs. 8 a–c), but comparison with the silymarin+LPS/D-GalN group showed no significant differences (Figs. 8 a–c).

**Fig. 8:** Treatment with SSB extract increased the expression levels of miR-124 in LPS/D-GalN-induced acute liver injury in mice. 24 h after the administration of LPS/D-GalN plus SSB extract, the miR-124 expression in LPS/D-GalN-induced mouse liver was determined via RT-PCR and in situ hybridization. **a** Representative in situ hybridization showing the level of miR-124 expression in liver tissue 24 h after the administration of LPS/D-GalN plus SSB. **b–c**: Representative RT-PCR and statistical summary of the densitometric analysis of miR-124 expression in the liver tissue 24 h after the administration of LPS/D-GalN plus SSB extract. Data are expressed as the mean ± SD. *P < 0.05: compared with the control group; #*P* < 0.05 and ##*P* < 0.01: compared with the model group. *P* > 0.05: control group compared with the control treatment group

RETRACTED

### Effects of SSB extract on hedgehog, Ptch, Smo, Gli, P13k, and Akt protein and gene expression levels in LPS/D-GalN-induced acute liver injury in mice

Hedgehog and P13k/Akt are important pathways for LPS/D-GalN-induced inflammation-related liver injury [29]. To observe the effects of SSB extract on Hedgehog, Ptch, Smo, Gli, P13k, and Akt protein and gene expression levels in LPS/D-GalN-induced mouse liver tissue, their gene and protein expression levels were determined via RT-PCR and Western blot analysis. As shown in Fig. 9, treatment with LPS/D-GalN significantly elevated the Hedgehog, Ptch, Smo, Gli, P13k, and Akt gene and Hedgehog, Ptch, Smo, Gli, P13k, and p-Akt protein expression levels compared with those of the control group. However, the Hedgehog, Ptch, Smo, Gli, P13k, and Akt gene and Hedgehog, Ptch, Smo, Gli, P13k, and p-Akt protein expression levels in the model SSB treatment group were significantly lower than those in the model group (Figs. 9 a–e). Comparison with the silymarin+LPS/D-GalN group showed no significant differences (Figs. 9 a–e).

**Fig. 9:** Effects of SSB extract on liver Hedgehog, Ptch, Smo, Gli, P13k, and Akt protein and gene expression levels in mice with LPS/D-GalN-induced acute liver injury. **a–b** Representative RT-PCR showing Hedgehog, Ptch, Smo, Gli, P13k, and Akt gene expression levels in liver tissue 24 h after the administration of LPS/D-GalN plus SSB extract. **c–d** Representative Western blot analysis showing Hedgehog, Ptch, Smo, Gli, P13k, and Akt protein expression levels in liver tissue 24 h after the administration of LPS/D-GalN plus SSB extract. **e** Statistical summary of densitometric analysis of Hedgehog, Ptch, Smo, Gli, P13k, and Akt protein expression in mouse liver tissue 24 h after the administration of LPS/D-GalN plus SSB extract. Data are expressed as mean ± SD. **P < 0.01: compared with the control group; #*P* < 0.05 and ##*P* < 0.01: compared with the model group. *P* > 0.05: control group compared with the control treatment group

### Effects of SSB extract on HMGB1, TRAF6, TLR4, IκB, p-IκB-α, and NF-κB65 protein expression in LPS/D-GalN-induced acute liver injury in mice

HMGB1/TLR4/NF-κB65 is a crucial inflammatory pathway that may be involved in LPS/D-GalN-induced acute liver injury [31]. We explored the effects of SSB extract on HMGB1, TRAF6, TLR4, IκB, p-IκB-α, and NF-κB65 protein expression in LPS/D-GalN-induced acute liver injury in mice. The HMGB1, TRAF6, TLR4, IκB, p-IκB-α, and NF-κB65 protein expression levels in mouse liver were determined via Western blot analysis. As shown in Fig. 10, the HMGB1, TRAF6, TLR4, p-IκB-α, and NF-κB65 protein expression levels significantly increased, and the IκB expression significantly decreased compared with that of the control group (Fig. 10 a and b). After treatment with SSB extract, HMGB1, TRAF6, TLR4, p-IκB-α, and NF-κB65 protein expression levels significantly decreased, and the IκB expression significantly increased compared with that of the model group (Fig. 10 a and b). Comparison with the silymarin+LPS/D-GalN group showed no significant differences (Fig. 10 a and b).

RETRACTED

**Fig. 10:** Effects of SSB extract on HMGB1, TRAF6, TLR4, IκB, p-IκB-α, and NF-κB65 protein expression, NF-κBp65 activity, and levels of DNA-bound NF-κB65 and TLR4 in LPS/D-GalN-induced acute liver injury in mice. **a** Representative Western blot showing HMGB1, TRAF6, TLR4, IκB, p-IκB-α, and NF-κB65 protein expression levels in mouse liver tissue 24 h after the administration of LPS/D-GalN plus SSB extract. **b** Statistical summary of the densitometric analysis of HMGB1, TRAF6, TLR4, IκB, p-IκB-α, and NF-kB65 protein expression levels in mouse liver tissue 24 h after the administration of LPS/D-GalN plus SSB extract. **e** and **f** Levels of DNA-bound NF-κB65 and TLR4 in mouse liver 24 h after the administration of LPS/D-GalN plus SSB extract. Data are expressed as mean ± SD. **P < 0.01: compared with the control group; #*P* < 0.05 and ##*P* < 0.01: compared with the model group. *P* > 0.05: control group compared with the control treatment group

### Effects of SSB extract on TLR4 and NF-κBp65 activity and levels of DNA-bound NF-KB65 and TLR4 in LPS/D-GalN-induced acute liver injury in mice

The levels of DNA-bound NF-KB65 and TLR4 play an important role in inflammatory transcription [29]. To investigate the effects of SSB extract on the levels of DNA-bound NF-κB65 and TLR4 in LPS/D-GalN-induced mouse liver, the NF-κBp65 activity and levels of DNA-bound NF-κB65 and TLR4 were determined. As shown in Fig. 10, the levels of DNA-bound NF-κB65 and TLR4 in LPS/D-GalN-induced mouse liver significantly increased compared with those of the control group (Fig. 10 c and d). However, after SSB extraction, the levels of DNA-bound NF-κB65 and TLR4 in LPS/D-GalN-induced mouse liver became significantly lower than those in the model group (Fig. 10 c and d). Comparison with the silymarin+LPS/D-GalN group showed no significant differences (Fig. 10 c and d).

### Effects of SSB extract on NF-κBp65 and TLR4 activity in LPS/D-GalN-induced mouse liver

To analyze the effects of SSB extract on NF-κBp65 and TLR4 activity in LPS/D-GalN-induced mouse liver, NF-κBp65 and TLR4 activities were measured via immunohistochemistry (IHC). As shown in Fig. 11, the NF-κBp65 and TLR4 activities in LPS/D-GalN-induced mouse liver were significantly elevated compared with those in the control and control SSB groups. After treatment with SSB extract, the NF-κBp65 and TLR4 activities in the model mice significantly decreased (Figs. 11 a–d). Comparison with the silymarin+LPS/D-GalN group showed no significant differences (Figs. 11 a–d). The NF-κBp65 and TLR4 activities in the control and control SSB groups were unchanged (Figs. 11 a–d).

RETRACTED

**Fig. 11:** Treatment with SSB extract decreased NF-κBp65 and TLR4 activities in LPS/D-GalN-induced mouse liver. **a** and **b** Representative IHC analysis showing NF-κBp65 and TLR4 activities in liver tissue 24 h after the administration of LPS/D-GalN plus SSB extract. **c** and **d** Statistical summary of IHC of NF-κBp65 and TLR4 activity in mouse liver tissue 24 h after the administration of LPS/D-GalN plus SSB extract. Data are expressed as mean ± SD. **P < 0.01: compared with the control group; #*P* < 0.05 and ##*P* < 0.01: compared with the model group. *P* > 0.05: control group compared with the control treatment group

### SSB extract treatment decreased MPO expression in LPS/D-GalN-induced mouse livers

MPO is an important indicator of leukocyte infiltration in the liver tissue [30]. MPO activity was significantly elevated in the LPS/D-GalN-induced mouse liver (Fig. 12 a). However, treatment with SSB extract decreased the MPO activity compared with that in the control group (Fig. 12 a). Comparison with the silymarin+LPS/D-GalN group showed no significant differences (Fig. 12 a).

**Fig. 12:** SSB extract treatment attenuated the activity of MPO and systemic inflammation in LPS/D-GalN-induced acute liver injury in mice. 24 h after the administration of LPS/D-GalN plus SSB extract, the activity of (**a**) MPO in the mouse liver was measured. The serum levels of (**b**) IL-6, (**c**) TNF-α, (**d**) IL-12, (**e**) ICAM-1, and (**f**) CRP were determined using ELISA. Data are expressed as mean ± SD. **P < 0.01: compared with the control group; #*P* < 0.05 and ##*P* < 0.01: compared with the model group

### Effect of SSB extract treatment on the serum levels of IL-6, TNF-а, CRP, IL-12, and ICAM-1 after LPS/D-GalN-induced acute liver injury in mice

IL-6, TNF-α, CRP, IL-12, and ICAM-1 are important inflammatory mediators in LPS/D-GalN-induced acute liver injury [32]. The serum levels of IL-6, TNF-α, CRP, IL-12, and ICAM-1 were determined using ELISA. As shown in Fig. 12, after LPS/D-GalN-induced acute liver injury in mice, the serum levels of IL-6, TNF-α, CRP, IL-12, and ICAM-1 were significantly increased (Figs. 12 b–f). However, after SSB extract treatment, the expression levels of IL-6, TNF-α, CRP, IL-12, and ICAM-1 in the serum significantly decreased (Figs. 12 b–f). Comparison with the silymarin+LPS/D-GalN group revealed no significant differences (Figs. 12 b–f).

RETRACTED

### Effects of SSB extract on serum ALT and AST and liver histology in LPS/D-GalN-induced acute liver injury in mice

ALT and AST are markers of hepatic damage [32]. To analyze the effects of SSB extract on serum ALT and AST and liver histology in LPS/D-GalN-induced acute liver injury in mice, the expression levels of ALT and AST were measured, and HE staining was carried out. The histopathological findings are shown in Fig. 13 a and b. The liver tissue was histologically normal in the control group (Fig. 13 a). By contrast, substantial intracellular vacuolization, sinusoidal dilatation, congestion, and focal necrosis of the liver parenchyma were observed in the LPS/D-GalN-induced group (Fig. 13 a). These changes decreased notably after SSB extract was administered in the treatment group, and the levels of substantial intracellular vacuolization, sinusoidal dilatation, congestion, and focal necrosis of the liver parenchyma in the treatment group were significantly improved compared with those in the model group (Fig. 13 a). The liver injury scores and serum levels of ALT and AST differed significantly between the model and model SSB groups (*P* < 0.0001; Figs. 13 b–d). This result indicates that pretreatment with SSB extract ameliorated LPS/D-GalN-induced histological changes. Comparison with the silymarin+LPS/D-GalN group revealed no significant differences (Figs. 13 a–d).

**Fig. 13:** Effects of SSB extract on ALT, AST, and liver histology in LPS/D-GalN-induced acute liver injury in mice. **a** HE-stained histology of rat liver tissue 24 h after the administration of LPS/D-GalN plus SSB extract. **b** Liver histology damage scoring (Suzuki score) from the four experimental groups 24 h after the administration of LPS/D-GalN plus SSB extract. **c** and **d** Levels of serum ALT and AST from the four experimental groups 24 h after the administration of LPS/D-GalN plus SSB extract

### Effects of SSB extract on the survival rate of mice with LPS/D-GalN-induced acute liver injury

The survival rate of mice with LPS/D-GalN-induced acute liver injury was significantly reduced compared with that of the mice in the control group. The decrement in the survival rate of mice with LPS/D-GalN-induced acute liver injury was significantly attenuated by pretreatment with SSB extract compared with that in the LPS/D-GalN-induced acute liver injury group. Comparison with the silymarin+LPS/D-GalN group revealed no significant differences (Fig. 14). After 96 h, survival rates of mice treated with SSB extract were higher than those treated with silymarin, but there was no statistical difference between the two groups (Fig. 14).

RETRACTED

**Fig. 14:** Treatment with SSB extract increased the survival rate of mice with LPS/D-GalN-induced acute liver injury. 120 h after the administration of LPS/D-GalN plus SSB extract, the survival rate of mice with LPS/D-GalN-induced acute liver injury was determined. Data are expressed as mean ± SD. **P < 0.01: compared with the control group; #*P* < 0.05 and ##*P* < 0.01: compared with the model group; *P* > 0.05: control group compared with the control treatment group

### Effect of quercetin, kaempferide, and isorhamnetin on cell proliferation inhibition rate in rat hepatocyte–KCs

To investigate the effect of active ingredients of SSB extract (quercetin, kaempferide, and isorhamnetin) on LPS-induced rat hepatocyte–KC inflammation and cell proliferation inhibition rate, hepatocyte–KCs were respectively incubated at various concentrations of quercetin, kaempferide, and isorhamnetin (25, 50, and 100 μg/ml) and LPS (1 mg/l) for 24 H*. IL*-6 and TNF-α in the hepatocyte–KCs were measured using ELISA, and cells proliferation inhibition rate was measured using MTT, As shown in Table 4, the quercetin, kaempferide, and isorhamnetin increased LPS-induced hepatocyte–KCs proliferation inhibition rate, and decreased the levels of IL-6 and TNF-α in the LPS-induced hepatocyte–KCs in a concentration-dependent manner (Figs. 7 a–b). Quercetin, kaempferide, and isorhamnetin concentrations as low as 50 μg/ml effectively decreased the IL-6 and TNF-α levels in the LPS-induced hepatocyte–KCs.

**Table 4:** Effect of quercetin, kaempferide, and isorhamnetin on cell proliferation inhibition rate in rat hepatocyte–KCs. The hepatocyte–KCs were respectively incubated at various concentrations of quercetin, kaempferide, and isorhamnetin (25, 50, and 100 μg/ml) and LPS (1 mg/l) for 24 H*. IL*-6 and TNF-α in the hepatocyte–KCs were measured using ELISA, and cells proliferation inhibition rate was measured using MTT. #*P* < 0.05: compared with the control group; *P < 0.05: compared with the LPS group

Drug	LPS (1 mg/l)	Dose (μg/ml)	Proliferation inhibition rate (%)	IL-6 (pg/ml)	TNF-α (pg/ml)
Control	**–**	**0**	**47.4 ± 10.4**	**0.43 ± 0.17**	**0.35 ± 0.11**
Model	+	**0**	**16.3 ± 4.6**^**#**^	**1.59 ± 0.64**^**#**^	**1.37 ± 0.37**^**#**^
Quercetin	+	**25**	28.6 ± 5.3*	0.98 ± 0.42*	0.84 ± 0.38*
	+	**50**	34.2 ± 7.1*	0.65 ± 0.29*	0.63 ± 0.19*
	+	**100**	43.8 ± 9.7*	0.49 ± 0.18*	0.48 ± 0.14*
kaempferide	+	**25**	**19.7 ± 7.9**	**1.33 ± 0.47**	**1.28 ± 0.41**
	+	**50**	31.1 ± 6.8*	0.85 ± 0.36*	0.89 ± 0.34*
	+	**100**	39.9 ± 11.7*	0.61 ± 0.19*	0.67 ± 0.22*
Isorhamnetin	+	**25**	**18.5 ± 8.2**	**1.37 ± 0.44**	**1.23 ± 0.47**
	+	**50**	31.9 ± 9.8*	0.89 ± 0.25*	0.92 ± 0.33*
	+	**100**	40.4 ± 11.3*	0.64 ± 0.18*	0.71 ± 0.29*

RETRACTED

## Discussion

Many treatments for liver injury are available. Liver transplantation therapy is limited by the age of the patient, insufficient supply of donors with the same human leukocyte antigen, multiple complications (e.g., infection), difficulty in the treatment of graft-versus-host disease, and high mortality rate. Drug treatment for acute liver injury is expensive, not remarkably effective, and has many toxic side effects. In this experiment, ALT and AST, focal and patchy necrosis in hepatic lobules, inflammatory cell infiltration, and acute liver injury score were significantly decreased after SSB extract was administered. Acute liver injury was significantly alleviated, and the survival rate of the mice increased. Studies have shown that SS can prevent the occurrence of D-GalN/LPS-induced acute liver injury by regulating anti-inflammatory and anti-apoptosis mechanisms [33, 34], but the specific mechanism is unclear. Therefore, we further explored the protective mechanisms of SS extract on LPS and D-GalN-induced acute liver injury.

In this experiment, a model of acute liver injury was established via intraperitoneal injection of D-Gal combined with LPS. After LPS/D-GalN intraperitoneal injection, the MPO activity in the liver tissue increased. Moreover, the inflammatory cell infiltration, the plasma levels of IL-6, TNF-α, CRP, and IL-12, and the production of inflammatory mediators and inflammatory markers increased. Intrahepatic and systemic inflammatory responses, AST and ALT, liver injury scores, and liver damage also markedly increased. Pathological HE staining showed that the structure of the hepatic lobule was blurred, the hepatic cells were disordered, the liver cells exhibited extensive cell degeneration, and obvious edema and balloon-like changes occurred. Focal and patchy necrosis was observed in the hepatic lobules. Moreover, central hepatic vein and hepatic sinus congestion was noted with increased inflammatory cell infiltration and high mortality rate, which are consistent with acute liver injury. After treatment with the SSB extract, the MPO activity in the liver tissue, inflammatory cell infiltration, and the levels of plasma IL-6, TNF-α, CRP, and IL-12 decreased. The production of inflammatory mediators and inflammatory markers was reduced, and the intrahepatic and systemic inflammation response was relieved. In addition, liver markers AST and ALT significantly decreased. The liver injury scores were reduced, liver damage was alleviated, and pathological HE staining showed that most liver cells were structurally intact and orderly arranged. Hepatocyte degeneration and necrosis were rarely observed, and the large patchy necrosis of hepatocytes was markedly relieved. A few mononuclear cells were infiltrated, showing an increased survival rate. These results suggest that the SSB extract might have exerted a protective effect on acute liver injury induced by LPS/D-GalN intraperitoneal injection.

miR-124 is an important inflammation-related miRNA. It can inhibit TRAF6 and IRAK1 in the TLR pathway and the activation of downstream NF-κB, thus playing anti-inflammatory roles [6]. We found that increasing the expression of miR-124 in rat hepatocyte–KCs could inhibit the activities of Hedgehog and P13k/Akt pathways and reduce the activity of the NF-κB/IκB pathway and the production of inflammatory mediators IL-6 and TNF-α. By contrast, inhibiting the expression of miR-124 in the rat hepatocyte–KCs could increase the activities of Hedgehog and P13k/Akt pathways, further stimulating the activity of the NF-κB/IκB pathway and increasing the production of inflammatory mediators IL-6 and TNF-α. miR-124 may regulate the activity of the NF-κB/IκB inflammatory pathway and inflammation in rat hepatocyte–KCs by regulating the Hedgehog pathway. Animal studies have found that in LPS- and D-GalN-induced rat liver tissues, the expression of miR-124 is significantly reduced, and the activities of Hedgehog and P13k/Akt pathways in the liver are increased. These phenomena stimulate the activity of the liver pro-inflammatory pathway. The inflammatory cells in the liver are increased, and liver damage is aggravated. After increasing the expression of miR-124 in the liver via intravenous injection of 1 × 10^9^ pfu AdCMV-miR-124, the activities of Hedgehog and P13k/Akt pathways in the liver were inhibited, the activity of the pro-inflammatory pathway was decreased, and LPS/D-GalN-induced acute liver injury was improved. Further studies showed that the SSB extract could significantly increase the expression of miR-124 in LPS/D-GalN-induced acute liver injury and reduce the inflammatory cells.

RETRACTED

When body tissues or cells are invaded by infectious or neoplastic factors, the inflammatory response and immune regulation of the body are activated by external stimulation and environmental stresses. The development-related Hedgehog signaling pathway is involved in the regulation of immune and inflammatory responses [35–37]. In the current study, LPS/D-GalN-induced liver tissues showed increased activity of the Hedgehog signaling pathway, increased expression of Ptch, Smo, and Gli genes and proteins, increased inflammation in the liver, and aggravated liver injury. In the LPS/D-GalN-induced liver tissues, treatment with SSB extract could significantly increase the activity of the Hedgehog signaling pathway, decrease the gene and protein expression levels of Ptch, Smo, and Gli, decrease the inflammatory cells in the liver, reduce the inflammation in the liver, and significantly decrease the liver injury.

We further explored the potential link between miR-124 and Hedgehog. Online Target Scan predicted that miR-124 binds with Hedgehog 3′-UTR. The luciferase reporter assay further demonstrated that Hedgehog is a target gene of miR-124. The present study is the first to identify the target relationship between Hedgehog and miR-124 and reveals that miR-124 mediates the mechanism of LPS/D-GalN-induced liver injury by regulating the Hedgehog expression. This finding suggests that Hedgehog can mediate its pro-inflammatory effects through the induction of miR-124. Therefore, SSB extract can reduce the activity of the Hedgehog signaling pathway by regulating the expression of miR-124 to reduce inflammation in the liver and protect the liver from injury induced by LPS and D-GalN. Studies have shown that the Hedgehog signaling pathway can activate the P13K/Akt pathway. P13K and its downstream molecule Akt are involved in NF-kB activity regulation, and they activate nuclear transcription factors, such as NF-kB, promote the production of several pro-inflammatory cytokines [34, 38], and induce or sustain inflammation [6]. In the present study, LPS/D-GalN-induced liver tissues showed increased activity of the Hedgehog signaling pathway, which activated the P13K/Akt pathway, leading to increased liver injury and liver inflammation. The administration of SSB extract blocked the activity of the Hedgehog signaling pathway, inhibited the P13K/Akt pathway, and alleviated liver injury and inflammation.

The occurrence and development of acute liver injury are closely related with the activation of HMGB1, which can cause the excessive release of inflammatory mediators by triggering the downstream TLR4/NF-κB signaling pathway [34], leading to liver injury. miR-124 can transregulate the activity of HMGB1/TLR4/NF-κB inflammatory pathways [39]. In the current study, the SSB extract increased the expression level of miR-124, inhibited the activity of the HMGB1/TLR4/NF-κB pathway, and reduced the inflammatory injury of the liver.

SS is rich in various chemical constituents, such as *Scutellaria*, flavonoids, triterpenoids, and alkaloids [40]. Studies have shown that the total flavonoids of SS are an important active component of hepatoprotective action in *Sedum sarmentosum*. The main active ingredients of total flavonoids of SS include quercetin, kaempferol, and luteolin. In this study, the HPLC analysis indicated that 1 g of SSB contained 0.93 mg of quercetin, 0.34 mg of kaempferide, and 0.27 mg of isorhamnetin, indicating that quercetin was the major component (Fig. 1). In this experiment, quercetin, kaempferide, and isorhamnetin effectively increased LPS induced rat hepatocyte–KCs proliferation inhibition rate, attenuated the production of IL-6 and TNF-α in the hepatocyte–KCs (Table 4). SSB extract concentrations effectively increased the miR-124 expression and blocked the activity of miR-124/Hedgehog and NF-κB65 signaling pathways in LPS-induced hepatocyte–KCs, SSB extract exhibits a protective effect on LPS and D-GalN-induced acute liver injury induced by regulating the proinflammatory pathways and proinflammatory mediators.

RETRACTED

Silymarin is a polyphenolic component isolated from the fruits and seeds of the milk thistle plant *Silybum marianum* (Asteraceae family) [41]. Silymarin extract contains approximately 65–80% flavonolignans (silybin A, silybin B isosilybin A, isosilybin B, silychristin, and silydianin), a small proportion of flavonoids, and approximately 20–35% fatty acids and polyphenolic compounds that possess a range of metabolic regulatory effects [42]. The hepatoprotective properties of silymarin in APAP intoxication have been previously described [41–45]. Silymarin extract exerted a protective effect on LPS and D-GalN-induced acute liver injury induced by regulating the proinflammatory pathways and proinflammatory mediators. Comparison with the SSB + LPS/D-GalN group revealed no significant differences.

## Conclusion

By increasing the expression levels of miR-124, the SSB extract could block the activity of the intracellular Hedgehog signaling pathway, inhibit the activities of the P13K/Akt and HMGB1/TLR4/NF-κB inflammatory pathways, and reduce liver inflammation and liver injury. This study revealed the protective mechanism of SSB extract in the treatment of acute liver injury and confirmed that Hedgehog is the inflammatory regulatory target of miR-124.

## Supplementary information

**Additional file 1: Table S1.** Treatment with SSB extract increased the survival rate of mice with LPS/D-GalN-induced acute liver injury. 120 h after the administration of LPS/D-GalN plus SSB extract, the survival rate of mice with LPS/D-GalN-induced acute liver injury was determined. Data are expressed as mean ± SD. **P < 0.01: compared with the control group; #*P* < 0.05 and ##*P* < 0.01: compared with the model group; *P* > 0.05: control group compared with the control treatment group. **Figure S1.** Treatment with SSB extract increased the survival rate of mice with LPS/D-GalN-induced acute liver injury. 120 h after the administration of LPS/D-GalN plus SSB extract, the survival rate of mice with LPS/D-GalN-induced acute liver injury was determined. Data are expressed as mean ± SD. **P < 0.01: compared with the control group; #*P* < 0.05 and ##*P* < 0.01: compared with the model group; *P* > 0.05: control group compared with the control treatment group. **Table S1** and **Fig. S1.** The survival rate of mice before revision. **Table S2.** same as table S1. **P < 0.01: compared with the control group; #*P* < 0.05 and ##*P* < 0.01: compared with the model group; *P* > 0.05: control group compared with the control treatment group. **Figure S2.** same as Figure S1. **P < 0.01: compared with the control group; #*P* < 0.05 and ##*P* < 0.01: compared with the model group; *P* > 0.05: control group compared with the control treatment group. **Table S2** and **Fig. S2.** The survival rate of mice after revision.

RETRACTED

## Data Availability

The datasets used and/or analyzed in the study can be made available by the corresponding author upon reasonable request.

## Abbreviations

Akt: Protein kinase B
D-GalN: D-galactosamine
HMGB1: High mobility group box 1
HPLC: High-performance liquid chromatography
LPS: Lipopolysaccharide
miR-124: microRNA-124
MPO: Myeloperoxidase
NF-κB: Nuclear factor kappa
SSB extract: *Sedum sarmentosum* Bunge extract
TLR4: Toll like receptor 4
